This article has been retracted.

# Does changing from a first generation antipsychotic (perphenazin) to a second generation antipsychotic (risperidone) alter brain activation and motor activity? A case report

**DOI:** 10.1186/1756-0500-6-182

**Published:** 2013-05-06

**Authors:** Jan Øystein Berle, Else-Marie Løberg, Ole Bernt Fasmer

**Affiliations:** 1 Division of Psychiatry, Haukeland University Hospital, Bergen, Norway; 2 Department of Biological and Medical Psychology, University of Bergen, Bergen, Norway; 3 Department of Clinical Medicine, Section for Psychiatry, Faculty of Medicine and Dentistry, University of Bergen, Bergen, Norway; 4 K way

**Keywords:** Schizophrenia, Antipsychotic, Brain activation, fMRI, Neurocognitive, Motor activity

## Abstract

**Background:**

In patients with schizophrenia, altered brain activation and motor activity levels are central features, reflecting cognitive impairments and negative symptoms, respectively. Newer studies using nonlinear methods have addressed the severe disturbances in neurocognitive functioning that is regarded as one of the core features of schizophrenia. Our aim was to compare brain activation and motor activity in a patient during pharmacological treatment that was switched from a first- to a second-generation antipsychotic drug. We hypothesised that this change of medication would increase level of responding in both measures.

**Case presentation:**

We present the case of a 53-year-old male with onset of severe mental illness in adolescence, ICD-10 diagnosed as schizophrenia of paranoid type, chronic form. We compared brain activation and motor activity in this patient during pharmacological treatment with a first-generation (perphenazin), and later switched to a second-generation (risperidone) antipsychotic drug. We used functional magnetic resonance imaging (fMRI) to measure brain activation and wrist worn actigraphy to measure motor activity.

**Conclusion:**

Our study showed that brain activation decreased in areas critical for cognitive functioning in this patient, when changing from a first to a second generation antipsychotic drug. However the mean motor activity level was unchanged, although risperidone reduced variability, particularly short-term variability from minute to minute. Compared to the results from previous studies, the present findings indicate that changing to a second-generation antipsychotic alters variability measures towards that seen in a control group, but with reduced brain activation, which was an unexpected finding.

## Background

Altered brain activation and reduced motor activity levels are central features of schizophrenia. Altered brain activation has often been reported in frontal regions during cognitive demanding tasks [1,2]. The term hypofrontality has been used by several authors to define this effect, which also has been seen in first-episode patients with schizophrenia [2] and neuroleptic-naive patients [1]. Recent studies present however a more complex picture, including for instance compensatory increased activation in other brain regions [1], altered brain activation in schizophrenia is seen as a reflection of the cognitive impairments in this patient group [2]. Cognitive impairments with clinical consequences are seen in a majority of patients with schizophrenia [3,4].

Reduced motor activity is one of several negative symptoms in schizophrenia. Motor retardation can be described as a reduction in motor activity as reflected in slowing or retardation of movements and speech, and reduced body tone. In addition, side-effects of the motor type are commonly reported when treating these disorders with antipsychotic medication [5], particularly when using first generation antipsychotics (FGA). Furthermore, a relationship between hypofrontality and physical anhedonia in schizophrenia has been reported [6]. Both cognitive impairments and negative symptoms have been shown to be important prognostic predictors in schizophrenia, predicting functional outcome better than positive symptoms [3,7].

It would be of clinical importance if there was a difference between a first-generation antipsychotic (FGA) and a second-generation antipsychotic (SGA) drug with regard to brain activation and motor activity. SGAs are hypothesized as having a more beneficial influence on the negative symptoms than the older (FGA) antipsychotics. The SGAs also have different pharmacological profiles with regard to brain regions involved in cognition and movement.

Thus, although functional neuroimaging traditionally is a research tool, studies of brain activation and motor activity may also have clinical consequences, on an individual level where there is a need for objective measures. The brain imaging method fMRI is a technique that allows detection of the brain areas that are involved in the performance of a cognitive or emotional task. We chose an arithmetic task with working memory load as the stimulus, or task, paradigm to tap cognitive processes attributed to frontal brain areas and brain areas rich in dopaminergic receptors [8], which could reflect effects of medication. The task was similar to the experimental design used by Hugdahl et al. [9].

Assessment of motor activity in psychiatry is seldom done using objective methods, in contrast to for example in neurology. In our study motor activity was monitored by a wrist worn actigraph. Actigraphy is an objective method to register accumulated motor activity over time for later analysis of movement frequency and amplitude. In schizophrenia, actigraphy has been used to investigate activity levels and circadian rest-activity phases and motor activity pattern [10,11].

The aim of our study was to explore putative changes in brain activation and in motor activity in a patient with schizophrenia during antipsychotic treatment with the FGA perphenazine and after switching to the SGA risperidone. We hypothesised that this change of medication would increase brain activation and motor activity.

## Case presentation

### The patient

The patients was male, Caucasian, and 53 years old. There were numerous incidences of severe mental illness in his family. His intellectual level was within the normal range; basic education, but no training or education as skilled worker or to a higher level. He had no significant somatic illness nor brain damage or other injuries. His alcohol consumption was within acceptable levels in the population and no use of illegal drugs was reported. This patient had symptom onset of severe mental illness in young adulthood; paranoid psychotic symptoms, auditory hallucinations, episodes with aggressive behaviour, dysfunction in activities of daily living. He was diagnosed with schizophrenia, paranoid type, chronic form, chronic phase (F20.0 in the ICD-10), although in periods affective symptoms of depression were present as well.

### Methods

In the first registration period the patient was treated with perphenazine decanoate 216 mg im/14th day, and in addition received chlorprotixene 100 mg and valproate 1200 mg daily. Drug monitoring revealed a trough serum level of perphenazine of 22 nmol/L, well above the recommended reference range of 1 to 6 nmol/L. Serum valproate was 467 nmol/L.

In the second registration period the antipsychotic medication was switched into risperidone (Risperdal Consta®), a long-acting intramuscular formulation. Drug monitoring of risperidone (s-risperidone + 9-OH risperidone) revealed a trough serum level of 114 nmol/L, serum level within the recommended reference range. Genotyping revealed that the patient was a CYP2D6 slow metabolizer (CYP2D6*4/CYP2D6*4).

The fMRI image acquisitions were done both during treatment with FGA, and again at follow-up ~6 months after the patient had been switched to a SGA. Cognitive function was examined using a mental arithmetic and working memory task where the patient had to add two-and-two successive numbers presented visually in LCD goggles, and press a response button placed on the chest whenever the sum of the numbers seen in the goggles was 10 [Figure 1]. fMRI was performed with a 1.5 T Siemens Vision Plus scanner equipped with 25 mT/m gradients. Initial scanning of anatomy was done with a T1W 3D FLASH pulse sequence. Thereafter, serial imaging with 100 BOLD sensitive echo planar (EPI pulse sequence) whole brain measurements were done during the task. Each EPI volume measurement consisted of 40 axial slices which constituted an image volume (FA/TA/TE/FOV/matrix = 50^0^/6 s/84 ms/230 mm/64×64). The in-plane pixel size was 3.44 × 3.44 mm, each slice with a thickness of 3.0 mm, thus creating nearly isotropic voxels. The first 10 image volumes were discarded prior to statistical analyses, to avoid artifacts due to stimulus novelty.

**Figure 1:** Task performed during the fMRI recordings.

There were 3 ON and 3 OFF blocks during task performance, presented in a box-car design. The digit stimuli were the numbers “1” through “9”. There were 16 trials with digit stimuli presented during each ON block, thus the total number of trials was 48. Each digit stimulus was presented for 300 ms, with 2200 ms blank interstimulus intervals (ISIs) in between. Thus, the total ON blocks lasted 120 sec, with a total of 60 sec OFF blocks. The ON and OFF blocks were alternated within the run. The digit stimuli were presented with the Micro Electronic Laboratory (MEL2) software (Psychology Software Tools Inc.). The OFF blocks consisted of resting with no stimulus presentations. The patient viewed the digit stimuli in electronic goggles consisting of a LCD-screen (Magnetic Resonance Technology Inc.) that were connected to a PC outside the MR chamber, which contained the MEL software. A response button was placed on the participant’s chest that he was instructed to press according to the specific instructions for each run. The patient was instructed to “add each consecutive number seen in the goggles to the previous one, and press the button whenever the sum was 10”. There were 6 presentations where the sum was “10” among the 16 trials for each ON block. Thus, the total number of target presentations, across the three ON blocks, were 18. The fMRI set-up was repeated twice in two separate sessions, with the different medications, respectively.

The fMRI images were statistically analyzed using the SPM5 software (http://www.fil.ion.ucl.ac.uk/spm). The data were first pre-processed, including realigning images, smoothing (8 mm) and normalizing to the standard MNI template and co-ordinate system, and then subjected to significance testing with t-tests.

Motor activity was monitored with an actigraph worn at the right wrist (Actiwatch, Cambridge Neurotechnology Ltd, England). The right wrist was chosen for the convenience of the participant. Previous studies have shown small differences between the right and left wrist. Total activity counts were recorded during one minute intervals. Motor activity was monitored on a 24 hour basis during two separate two week periods 6 months apart performed when the patient was on FGA (perphenazine), and later after switching to SGA (risperidone). The fMRI were performed in close proximity to these two periods.

Both medications were given as intramuscular depot injections to ensure adherence to treatment, and therapeutic drug monitoring (TDM) were performed on both medications to ensure adequate dosage. All samples were analyzed by a LC/MSD method. Genotyping of CYP2D6 was also performed to evaluate the patient’s metabolic capacity.

Average activity per minute, the standard deviation (SD), the root mean square successive differences (RMSSD), the relation between RMSSD and SD (RMSSD/SD), and sample entropy were calculated for one continuous activity period each day, defined as the longest period containing not more than 9 consecutive minutes with zero activity. These are the same mathemathical methods used in our previous studies [10,11]. Results are presented as mean ± SD for 21 periods during perphenazine treatment and 27 periods during risperidone treatment.

Sample entropy is a nonlinear measure, indicates the degree of regularity (complexity) of time series, and is the negative natural logarithm of an estimate of the conditional probability that subseries of a certain length (m) that match point-wise, within a tolerance (r), also match at the next point. For the present study m = 2 and r = 0.2 were chosen.

SPSS version 15.0 was used for the statistical analyses.

### Results

The results from the fMRI acquisition showed significant activations during the mental arithmetic task when analyzed separately for the two sessions (using an uncorrected significance threshold of p < .001), in the occipital lobe, right parietal lobule, and pre-central / SMA area, and in an extended area in the pre-motor areas in the frontal lobe (BA 4/6), and in the superior parietal lobule (BA7). The parietal activation for the mental arithmetic task would fit previous findings of parietal cortex activations for number calculations, in particular with a right-sided laterality effect. Figure 2 shows the difference activation between session 1 (FGA) and 2 (SGA).

**Figure 2:** fMRI results.

We also compared the activation in condition 2 (SGA) and condition 1 (FGA), by subtracting the images for the respective condition, using an uncorrected significance threshold of p < .01 due to loss of degrees of freedom. This showed remaining activations when subtracting images for condition 2 from images for condition 1 in the right inferior frontal/insula region, (BA 13) extending across the premotor cortex, in the superior parietal lobule (BA 7) and in the occipital lobe/lingual gyrus (BA 18). Increasing the significance threshold to p < .001 did not yield any significantly remaining effects for condition 1 compared to condition 2.

Results of the actigraph recordings are shown in Table 1. Mean daytime motor activity was not changed after switching of medication. The standard deviation was slightly, but not significantly, lower with risperidone than with perphenazine. The RMSSD however, was significantly reduced after switching to risperidone, and also the RMSSD/SD ratio.

**Table 1:** Results from actigraphic recordings (mean ± SD)

	**Perphenazin**	**Risperidone**
**Mean activity**	301 ± 79	298 ± 48
**SD**	270 ± 67	254 ± 43
**RMSSD**	250 ± 48	216 ± 19**
**RMSSD/SD**	0.94 ± 10	0.87 ± 12*
**Sample entropy**	1.35 ± 0.18	1.33 ± 0.29

* p <0.05 t-test.

** p <0.01 t-test.

## Conclusions

This study showed that brain activation decreased in areas critical for cognitive functioning, when a patient with schizophrenia was changed from FGA to a SGA medication. Total motor activity, however, was not altered during this change in medication, although our findings interestingly indicate that a change to SGA alters variability measures towards what was seen in a healthy control group shown in one of our prior studies [11].

We do not have test-retest data for fMRI from this particular study. This may represent a limitation of the study, since intra- and inter-individual variability generally is a problem in fMRI studies. However we do not think that our findings are caused by such confounding effects, since other studies, using variants of the same paradigm have shown similar patterns as found after medication in the present study [9,12]. An additional limitation of the fMRI data is the possibility that some of the changes from the first to the second session could be driven by learning effects and by the instruction to press the response button on target trials, which could lead to reduced activation due to facilitation. This is however not likely to explain all the findings that also were outside of areas to be affected. Another limitation is the rather weak statistical effects, not surviving standard correction procedures for multiple significance tests. Such procedures are typically applied to group average data, and may have reduced applicability for a single case study.

A case study like the current study has its obvious limitations when it comes to generalizations to the population of schizophrenia patients. However, group averages based on large samples could equally be criticised for lacking in representativeness for a single patient, which is what the clinician is facing. Group averages are by definition not fully representative for any individual subject in the group, both because of the effect of statistical averaging and from the perspective of individual variation in response to antipsychotic medication (which is substantial in schizophrenia). Thus, reporting data for a single patient, measured longitudinally, being his own control, may yield clinically relevant data.

The patterns of variability in the motor activity after switching antipsychotics from a FGA to a SGA are not easy to interpret. While the mean motor activity level and sample entropy were unchanged, risperidone reduced variability, particularly the variability from minute to minute, reflected in the RMSSD and also the RMSSD/SD ratio, towards what has been reported in healthy controls [11]. Nonlinear methods have addressed the severe disturbances in neurocognitive dysfunctioning as one of the core features of schizophrenia [13,14]. Wrist worn actigraphy for motor registration and magnetic resonance imaging for brain activation have shown correlations between motor activity and changes in brain structure [15]. Our findings comparing a patient switching from a first to a second generation antipsychotic supports these findings.

The high perphenazine level observed in our patient could be explained by the low CYP2D6 metabolic capacity [16].

The decreased activation in the right inferior frontal and insula region is somewhat of a puzzle since one would have expected increased activation. It has been suggested that the inferior frontal gyrus and anterior insula areas are involved in complex attentional and working memory processing. Possibly, these brain areas are involved in cognitive control related to attentional focus on stimuli that are urgent or close in time and space [17], and it is unclear how such functions relate to reduced activation. Moreover, the right fronto-insular cortex has been implicated in a wide range of cognitive control mechanisms involved in a variety of cognitive control processes, including conflict and error monitoring, interference resolution, and response selection [18]. The inferior frontal gyrus and anterior insula has also been associated with psychosis. Insular dysfunction may be important for the development of psychosis due to its influence on the salience network [19]. Furthermore, the right inferior frontal area and posterior insula has been indicated in auditory hallucinations [20].

We conclude that changes in neuronal brain activation decreased in areas critical for cognitive functioning when a patient with schizophrenia was changed from a FGA to a SGA. At the same time although the total motor activity was not altered, variability measures changed towards values seen in healthy controls. Our study underscores the value of casuistic reports of schizophrenic patients examined during different conditions using objective recording methods in pharmacological treatment studies. Although the actigraph data were partly in accordance with the hypothesis, the brain activation results were unexpected, and not hypothesized and would need careful replication in a group study with proper statistical power, before any firm conclusions can be reached.

## Consent

Written informed consent was obtained from the patient for publication of this Case report and any accompanying images. A copy of the written consent is available for review by the Editor-in-Chief of this journal.

## Competing interest

The authors declare that they have no competing interests.

## Authors’ contributions

JØB introduced the patient to this study. JØB and OBF made the motor activity measures. EML performed the cognitive investigations. All authors participated in its design and coordination and helped to draft the manuscript. All authors read and approved the final manuscript.
